# Painless Gastrointestinal Endoscopy Assisted with Computed Tomography Image Information Data Monitoring in Postoperative Neurocognitive Dysfunction in Patients with Combined Anesthesia of Propofol and Butorphanol Tartrate under Electronic Health

**DOI:** 10.1155/2022/7086472

**Published:** 2022-06-20

**Authors:** Yueguang Wei, Jianxun Liu, Xuhai Gong

**Affiliations:** ^1^Department of Gastroenterology, Daqing Oilfields General Hospital, Daqing, 163000 Heilongjiang, China; ^2^Department of Neurology, Daqing Oilfields General Hospital, Daqing, 163000 Heilongjiang, China

## Abstract

The aim of this study was to explore the value of computed tomography (CT) images based on electronic health (E-health) combined with painless gastrointestinal endoscopy (PGE) in the diagnosis of neurocognitive function in patients with combined anesthesia of propofol and butorphanol tartrate. 126 patients undergoing PGE were selected as the research objects, and all were performed with CT perfusion imaging before and after anesthesia to obtain the cerebral blood volume (CBV), cerebral blood flow (CBF), mean transit time (MTT), and time to peak (TTP). The Montreal Cognitive Assessment (MoCA) was adopted to evaluate the cognitive function of patients. The results showed that after anesthesia, the levels of CBF and CBV in the left and right thalami, frontal lobe, and temporal lobe of the patients were lower than those before anesthesia, while TTP and MTT were higher than those before anesthesia (*P* < 0.05). The MoCA score after anesthesia was lower than that before anesthesia (*P* < 0.05). After anesthesia, the CBF, CBV, TTP, and MTT values of the left and right frontal lobes and left and right temporal lobes were significantly positively correlated with MoCA (*P* < 0.05). In conclusion, the brain CT image parameters based on E-health can clearly display the blood perfusion in the lesion area of the patient, which was beneficial to the PGE-assisted judgment of cognitive dysfunction in patients with propofol tartrate and butorphanol tartrate anesthesia. Therefore, CT-assisted PGE examination based on E-health had a certain clinical value in evaluating the neurocognitive function of patients.

## 1. Introduction

Digestive endoscopy is to understand the pathological changes of the stomach and colon through gastroscopy and colonoscopy. It can examine the esophagus, stomach, and duodenum with a flexible tube endoscope through the mouth or anus to see if there is a tumor or ulcer or a card with something stuck in the esophagus or elsewhere [1, 2]. Most of the early gastrointestinal lesions are asymptomatic, so it is clinically recommended that men over the age of 40-45, especially those with a family history of tumors, undergo gastrointestinal endoscopy in a timely manner, so as to achieve early detection, early treatment, and early prevention of cancers [3]. Gastrointestinal endoscopy can be divided into two methods: general and anesthesia. The former can be achieved by oral lidocaine-type anesthetics, but patients may experience uncomfortable symptoms such as nausea and vomiting. The latter use analgesic and sedative drugs, which allow gastrointestinal endoscopy to be performed without causing any pain to the patient, and can be done during sleep [4, 5].

At present, deep sedation is often used for gastrointestinal endoscopy in the department of gastroenterology. Propofol is a commonly used drug for general anesthesia, induction, and maintenance. It can be used in combination with analgesics, muscle relaxants, and inhalation anesthetics, so it is suitable for outpatient use [6]. Butofino tartrate can interact with certain receptors in the central nervous system and indirectly exert analgesic effect, which is suitable for the treatment of various types of cancer pain and postoperative pain. Based on this, combined anesthesia of propofol and butofino tartrate was used in patients undergoing PGE examination [7]. However, it is clinically found that many patients have symptoms such as memory loss and emotional anxiety after painless gastrointestinal endoscopy (PGE) examination, so it has a great adverse effect on the cognitive function of patients. Therefore, this paper intends to explore the effect of PGE examination on neurocognitive function of patients under anesthesia.

With the advancement of imaging technology, computed tomography (CT) perfusion imaging has gradually developed on the basis of ordinary CT effects. It is different from dynamic scanning. Through rapid intravenous injection of contrast agent, continuous CT scanning is performed in the brain region of interest, and the time-dose curve (TDC) of the brain region of interest can be obtained, and then, the values of various perfusion parameters are calculated [8]. Currently, CT perfusion imaging is mainly used in the study of acute cerebral ischemia and tumors. In the case of cerebral ischemia, part of the blood flow is reduced, the degree of ischemia can be understood, and the hemodynamic changes of the unit tissue can be quantitatively analyzed by perfusion. In this way, the ischemic tissue can be evaluated, and normal blood supply can be restored in time. Tumor perfusion is to investigate the perfusion value and capillary permeability caused by neovascularization, thereby inhibiting tumor growth through antiangiogenesis [9–11]. In this work, CT perfusion imaging technology was used to analyze the images of patients with PGE.

In conclusion, patients who were anesthetized with propofol and butorphanol tartrate were selected as the research objects in this work. By using the E-health-based CT images, it explored the PGE examination under combined anesthesia with propofol and butnorphine tartrate and assessed the neurocognitive function of patients comprehensively. It was hoped that the evaluation of neurocognitive dysfunction in patients after anesthesia would provide some reference value.

## 2. Materials and Methods

### 2.1. Sample Selection

In this study, 126 patients enrolled in the PGE examination (combined anesthesia of propofol and butorphanol tartrate) in hospital from May 2019 to April 2020 were selected as research objects, including 72 males and 54 females, with an age range of 20-68 years. In terms of the age of the patients, the proportion of patients aged 40-50 was the highest (51 cases, 40.47%), followed by those over 50 years old (48 cases, 38.10%) and those under 40 years old (27 cases, 21.47%). Secondly, among all patients, the patients with hospitalization time of 3-5 months accounted for the highest proportion (40.48%), the patients with hospitalization time of more than 5 months accounted for 36.51%, and the patients with hospitalization time of less than 3 months accounted for 23.02%. In terms of disease reasons, the proportion of patients undergoing microscopic examination due to intestinal polypectomy was the highest (42.06%), followed by patients with gastric polypectomy (31.75%) and other reasons (26.19%). This study had been approved by ethics committee of hospital, and the patients and their families had signed the informed consents.

Inclusion criteria are as follows: patients with stable vital signs, patients older than 18 years of age, patients without CT-tested contraindications, and patients with complete clinical data.

Exclusion criteria are as follows: patients who could not complete the follow-up examinations for personal reasons, patients who have received related treatment, patients with combined mental disorders, patients with gastrointestinal endoscopy contraindications, and patients with major complications (cardiac arrest, haemorrhage, etc.).

### 2.2. Examination by Painless Gastrointestinal Endoscopy

The patient was required to fast for eight hours and no water for four hours and then take the appropriate amount of simethicone. The patient was required to sleep on the bed at a lateral position with knee bending, with bite block in the mouth. The patient was injected with intravenously 0.06 mg/mL of butorphanol tartrate and added with 2 mg/kg of propofol 2 minutes later. After the patient can take self-breathing smoothly, the gastroscopy examination was started. The trachea intubation, pressurized feeding equipment, and emergency medicine had to be prepared ready for emergency use.

### 2.3. Computed Tomography Perfusion Imaging

Patients were examined on a cross-sectional basis using 64 rows of 128-layer gem helical CT. Before the scan, the patient was placed in a supine position, with the head in the headrest. The patient was injected with 60 mL of iopromide injection and then performed with the CT perfusion imaging scanning at the standard level of the brain base section area for a total of 15 cycles to obtain the TDC. The scanning parameters were set as follows: tube voltage of 120 kV, automatic tube current, layer thickness of 10 mm, matrix of 512 × 512, and field of view 200 × 200 mm. After the scan was completed, the image was processed by using the stroke analysis software to obtain the values of CBV, CBF, MTT, and TTP in the thalamus, frontal lobe, parietal lobe, temporal lobe, and occipital lobe.

### 2.4. Patient Data Collection

The age, height, weight, gender, and hospital stay of all patients were recorded. Subjects were evaluated using the MoCA [12]. The CT perfusion imaging data of all patients were recorded.

### 2.5. Statistical Methods

The data processing was analyzed by the SPSS19.0 version statistical software, the measurement data was expressed by mean of standard deviation ($\overset{¯}{x}\pm s$), and the counting data was indicated as a percentage (%). The values of CBV, CBF, MTT, and TTP in the thalamus, frontal lobe, parietal lobe, temporal lobe, and occipital lobe of patients before and after anesthesia were compared with *t*-test. The scores of MoCA before and after anesthesia were compared with variance analysis. *P* < 0.05 indicated that there was a statistical significance.

## 3. Results

### 3.1. CT Image of Patient after Anesthesia

Figure 1 shows the images of routine CT examinations after anesthesia in several patients. In Figure 1(a), quasi-circular hypodense shadow with clear edges was seen in the left cerebellar hemisphere, and an epidural hyperdense shadow was found. It had mild signs and no obvious edema. In Figure 1(b), small patches of low-density shadows were found in the anterior horns on both sides, the left coronal radiating area was unclear, the fourth ventricle was slightly displaced due to certain pressure, the upper ventricle was dilated without obvious hydrops, and the left eyeball was calcification.  Figure 1(c) shows that the left temporal lobe and parietal lobe found stud-shaped density shadows with clear edges and uniform density. The corresponding ventricles were not clear, the left ventricle was slightly compressed, and the midline structure was slightly shifted to the right.

### 3.2. Comparison of Thalamus CT Parameters before and after Anesthesia

As shown in Figure 2, the levels of CBF, CBV, TTP, and MTT in the left thalamus of patients before anesthesia were 64.74 ± 9.31, 50.81 ± 6.08, 74.75 ± 9.24, and 98.47 ± 9.56, respectively; those in the right thalamus were 63.96 ± 6.84, 49.68 ± 5.24, 78.31 ± 5.62, and 86.92 ± 9.79, respectively; the levels of above four indicators in the left thalamus of patients after anesthesia were 45.84 ± 7.55, 38.86 ± 5.11, 113.62 ± 20.33, and 120.61 ± 12.43, respectively; the levels in the right thalamus after anesthesia were 48.07 ± 9.64, 35.92 ± 4.77, 108.47 ± 18.21, and 117.13 ± 11.78, respectively. Of which, the levels of CBF and CBV in both left and right thalami after anesthesia were significantly lower than those before anesthesia, and the differences were statistically significant (*P* < 0.05), and the levels of TTP and MTT in both sides after the anesthesia were higher observably than those before the anesthesia.  Figure 3 shows the CT perfusion imaging images for several patients and suggests clearly that the CBV and CBF were decreased and the TTP and MTT were increased.

### 3.3. Comparison of CT Parameters in the Frontal Lobe before and after Anesthesia

Figure 4 suggests that the level of CBF and CBV in the left and right frontal lobes after anesthesia was significantly lower than the levels before the anesthesia, and the difference was statistically significant (*P* < 0.05), while the level of TTP and MTT in the left and right frontal lobes after anesthesia was greatly higher than the levels before the anesthesia, and the difference was statistically significant (*P* < 0.05).

### 3.4. Comparison of CT Parameters in the Occipital Lobe before and after Anesthesia

Figure 5 reveals that the CBF in the left and right occipital lobes after anesthesia was significantly lower than that before anesthesia, and the difference was statistically significant (*P* < 0.05), while the level of CBV, TTP, and MTT was higher observably than those before the anesthesia, and it had no statistically significant difference (*P* > 0.05).

### 3.5. Comparison of CT Parameters in the Temporal Lobe before and after Anesthesia in Patients

As shown in Figure 6, the CBF and CBV in the left and right temporal lobes of the patient after anesthesia were significantly lower than those before anesthesia, and the difference was statistically significant (*P* < 0.05), while the TTP and MTT were higher obviously than those before the anesthesia with statistically significant difference (*P* < 0.05).

### 3.6. Comparison of MoCA Scores before and after Anesthesia

Figure 7 discloses that the MoCA score was 19.65 ± 6.21 before anesthesia, and the score of MoCA after the anesthesia was 26.82 ± 7.26, respectively. Of which, the MoCA score was significantly decreased after anesthesia with the difference of statistical significance (*P* < 0.05).

### 3.7. Analysis on the Correlation between CT Parameters and Scores

Table 1 discloses that the CBF, CBV, TTP, and MTT values in the left and right thalami have very obviously positive correlations with MoCA score (*P* < 001). The values of four indicators in the left and right frontal and temporal lobes have visibly positive correlations with MoCA score (*P* < 0.05). CBF value in the left and right occipital lobes was extremely, sharply, and positively correlated with MoCA score (*P* < 0.001), and the values of CBV, TTP, and MTT were not considerably correlated with both MoCA scores.

## 4. Discussion

With the development of endoscopy technology, the gastroscope and colonoscopy play very important roles in clinical diagnosis, can be used for the examination of all digestive tracts, and guide of related surgery, such as gastric polyp removal and stone removal. However, PGE requires propofol or other anesthetic drugs, which may affect the patient's neurocognitive function [13]. Based on this, patients undergoing PGE were scanned and examined with CT perfusion imaging, and it was found that the CBF and CBV levels in the left and right thalami after anesthesia were significantly decreased, while the TTP and MTT levels were greatly increased, and the differences were statistically significant (*P* < 0.05). Such results were similar to the results of Rodriguez et al. [14], which disclosed that CBF referred to the blood flow through a certain region of brain tissue blood vessels in a unit of time, so blood supply in the left and right thalami was insufficient and part of the brain tissue suffered incomplete cycle after the patients was narcotized. CBV can reflect the blood capacity of a certain region of brain tissue, and the decline of CBV means that the patient's vascular replacement capacity is reduced [15]. TTP refers to the time-to-peak of contrast agent in brain tissue, and it can reflect a decrease in cerebrovascular circulation resistance and insufficient early vascular perfusion. The CBF and CBV levels in the left and right frontal lobes after anesthesia were greatly decreased, and the TTP and MTT levels were increased obviously with the difference of statistical significance (*P* < 0.05), which also showed that the blood supply in the left and right frontal lobes after anesthesia was insufficient, part of brain tissue suffered incomplete cycle, and the blood vessel replacement ability was decreased [16]. The CBF and CBV levels in the left and right temporal lobes after anesthesia were decreased obviously, and the TTP and MTT levels were increased observably with the difference of statistical meaningfulness (*P* < 0.05). It was the same as the results of the left and right thalami and frontal lobe, which also showed that the patient suffered from insufficient blood supply in brain tissue after anesthesia.

In addition, it was found that the CBF level of the left and right side occipital lobe after anesthesia was significantly decreased, while the levels of CBV, TTP, and MTT were not statistically significant before and after anesthesia (*P* > 0.05), which differed from the results of the study of Xue et al. [17]. It may be that different brain tissue perfusion parameters had large differences in different brain regions, which were related to the different cognitive functions of the body that were regulated, but the specific internal connections had to be further explored [18]. The result revealed that the MoCA score after anesthesia was significantly decreased, and the differences were statistically significant (*P* < 0.05). It indicated that the patient's neurocognitive function decreased after anesthesia, and even permanent damage could be resulted in, thereby increasing the risk of treatment [19]. In order to further explore the correlation between CT perfusion parameters and the patient's neurocognitive function, Spearman correlation was adopted for analysis, and the results disclosed that CBF, CBV, TTP, and MTT values in the left and right thalami had very significantly positive correlations with the MoCA score (*P* < 0.001). The CBF, CBV, TTP, and MTT values in the left and right frontal and temporal lobes were observably and positively correlated with the MoCA score, and obviously (*P* < 0.05), which was similar to the above analysis results, indicating that CT perfusion imaging parameters CBF, CBV, TTP, and MTT can be undertaken as important indicators to reflect the neurocognitive dysfunction of patients and have certain degree of promotion value [20].

## 5. Conclusion

In this work, PGE based on CT image information was used to evaluate postoperative neurocognitive function of patients under propofol and butorphanol tartrate combined anesthesia. In addition, the correlations between such parameters and MoCA scores were analyzed. The results showed that the neurocognitive function declined in patients with PGE after anesthesia and the CBF, CBV, TTP, and MTT could be considered as important indicators to reflect the cognitive dysfunction of patients and had certain promotion value. However, the basic data of each patient was collected, but it did not analyze the effects of age, gender, propofol dosage, and other factors on the cognitive function of patients in PGE examination. Thus, it is considered increasing the sample size of patients in following researches. In summary, the results of this article provide an experimental basis for the judgment of neurocognitive dysfunction in patients with PGE examination (combined anesthesia of propofol and butorphanol tartrate).

## Figures and Tables

**Figure 1:** The images of routine CT examination after anesthesia of several patients. (a) showed the CT image of a male patient (aged 49 years old). (b) gave the CT image of a male patient (aged 65 years old). (c) revealed the CT image of a female patient (aged 53 years old).

**Figure 2:** Comparison of thalamus CT parameters before and after anesthesia. (a–d) showed the level of CBF, CBV, TTP, and MTT in the thalamus, respectively. ^∗^Compared with the levels before anesthesia, *P* < 0.05.

**Figure 3:** CT perfusion imaging images of patients. (a–d) disclosed the level of CBV, CBF, TTP, and MTT, respectively. White arrows pointed out the patient's focal area.

**Figure 4:** Comparison of CT parameters in the frontal lobe before and after anesthesia. (a–d) suggested the CBF, CBV, TTP, and MTT in the frontal lobe. ^∗^Compared with the level before anesthesia, *P* < 0.05.

**Figure 5:** Comparison of the CT parameters in the occipital lobe before and after anesthesia in patients. (a–d) illustrated the level of CBF, CBV, TTP, and MTT in the occipital lobe, respectively. ^∗^Compared with the level before anesthesia, *P* < 0.05.

**Figure 6:** Comparison of CT parameters in the temporal lobe before and after anesthesia. (a–d) were CBF, CBV, TTP, and MTT in the temporal lobe, respectively. ^∗^Compared with the level before anesthesia, *P* < 0.05.

**Figure 7:** Comparison of MoCA scores before and after anesthesia. ^∗^Comparing with the scores before anesthesia, *P* < 0.05.

**Table 1:** Analysis of the correlation between CT parameters and scores.

Brain area		MoCA
		*r*
Left thalamus	CBF	0.397^∗∗^
	CBV	0.462^∗∗^
	TTP	0.392^∗∗^
	MTT	0.418^∗∗^
Right thalamus	CBF	0.522^∗∗^
	CBV	0.388^∗∗^
	TTP	0.427^∗∗^
	MTT	0.511^∗∗^
Left frontal lobe	CBF	0.384^∗^
	CBV	0.326^∗^
	TTP	0.309^∗^
	MTT	0.413^∗^
Right frontal lobe	CBF	0.472^∗^
	CBV	0.385^∗^
	TTP	0.346^∗^
	MTT	0.428^∗^
Left occipital lobe	CBF	0.385^∗^
	CBV	0.144
	TTP	0.165
	MTT	0.227
Right occipital lobe	CBF	0.481^∗^
	CBV	0.194
	TTP	0.181
	MTT	0.252
Left temporal lobe	CBF	0.451^∗^
	CBV	0.332^∗^
	TTP	0.362^∗^
	MTT	0.401^∗^
Right temporal lobe	CBF	0.611^∗^
	CBV	0.372^∗^
	TTP	0.386^∗^
	MTT	0.521^∗^

^∗^ suggested *P* < 0.05. ^∗∗^ suggested *P* < 0.001.

## Data Availability

The data used to support the findings of this study are available from the corresponding author upon request.
